This article has been retracted.

# Influence of Gestational Hypertension on Cardiovascular Health Behaviors and Factors

**DOI:** 10.1155/2022/1031418

**Published:** 2022-03-29

**Authors:** Haiyan Zhao, Yuntao Wu, Junyan Sun, Changhao Zu, Chunyu Ruan, Kai Cui, Honghong He, Shouling Wu, Xiaojing Peng

**Affiliations:** ^1^Departments of Cardiology, Kailuan General Hospital, Tangshan 063000, Hebei, China; ^2^Departments of Anesthesiology, Kailuan General Hospital, Tangshan 063000, Hebei, China

## Abstract

**Objective:**

A survey was conducted to analyze the epidemiological differences in ideal cardiovascular health (CVH) behaviors and factors after delivery in females with and without gestational hypertension (GH) and evaluate the influence of GH on cardiovascular health behaviors and factors.

**Methods:**

The present study adopted a cross-sectional design. A total of 4620 female workers who gave birth between 1976 and 2012 and received the annual health examination (2012 to 2013) at hospitals belonging to the Kailuan Medical Group were recruited. These subjects were divided into the GH group and non-GH (NGH) group, depending on whether they were combined with GH or not at delivery. The epidemiological differences in CVH behaviors and factors were compared between the two groups.

**Result:**

In both groups, the percentage of subjects achieving ideal smoking status was the highest, while the percentage of subjects achieving an ideal level of physical activity was the lowest among all behaviors and factors. Compared with the NGH group, the percentages of subjects achieving each of the seven ideal CVH metrics decreased in the GH group. The percentages of subjects achieving ideal body mass index (BMI), blood pressure, blood glucose level, and cholesterol level were significantly lower in the GH group than in the NGH group (*P* < 0.05). The percentage of subjects with an ideal level of physical activity was higher in the NGH group than in the GH group. After stratification by age, the percentages of patients achieving ideal BMI, blood pressure, and blood glucose decreased with age regardless of the history of GH (*P* < 0.05). In the younger age group, the percentage of subjects with GH achieving ideal body mass index was significantly lower than that of those without GH.

**Conclusion:**

Compared with females without GH, those with GH had higher BMI, blood pressure, blood glucose level, and cholesterol level among the seven CVH metrics surveyed.

## 1. Introduction 

In the early 20^th^ century, the emerging fact that the mortality of cardiovascular diseases in females was higher than that of males began to attract attention. Since then, a greater emphasis has been placed on research on heart diseases in women. Efforts have been made to improve the treatment for heart diseases in women and narrow the gap in survival between females and males with heart diseases. Women shoulder the responsibility of bearing life and may encounter a higher risk of a premature initiation of maternal and infant cardiovascular and cerebrovascular diseases. A large number of studies have shown that compared with females without a history of gestational hypertension (GH), those with such a history are faced with aggregation of conventional cardiovascular risk factors [1–3] and a higher likelihood of early cardiovascular and cerebrovascular events in the long term [4–6]. GH may be an initiating factor for cardiovascular events in females. American Heart Association (AHA) has proposed the concept of cardiovascular health (CVH) behaviors and factors for the purpose of primary prevention [7]. Compared with healthy parturients, those with a history of GH may have different epidemiological characteristics of CVH behaviors and factors in the long term. The present study was concerned with the distribution of CVH behaviors and factors in females with and without GH after delivery.

Our contribution in this study is as follows:

1. To analyze the epidemiological differences in ideal cardiovascular health (CVH) behaviors
2. To also analyze factors after delivery in females with and without gestational hypertension (GH)
3. To evaluate the influence of GH on cardiovascular health behaviors and factors

## 2. Subjects and Methods

### 2.1. Subjects a Cross-Sectional Study Design Were Adopted

The subjects were selected according to the following criteria: (1) female workers giving birth at hospitals belonging to Kailuan Medical Group from October 1976 to December 2012 (including Kailuan Hospital, Kailuan Linxi Hospital, Kailuan Zhaogezhuang Hospital, Kailuan Fangezhuang Hospital, Kailuan Lvjiatuo Hospital, Kailuan Linnancang Hospital, Kailuan Majiagou Hospital, Kailuan Jingezhuang Hospital, Kailuan Tangjiazhuang Hospital, and Kailuan Qianying Hospital), with complete delivery records, (2) first singleton birth, (3) having received the annual physical examination for on-duty and retired staff at hospitals belonging to the Kailuan Medical Group from July 2012 to October 2013, and (4) having consented to participate in the present study and signed the informed consent form. The exclusion criteria were as follows: (1) having a prior history of hypertension before pregnancy, (2) induced or natural abortion, (3) secondary hypertension, and (4) incomplete research data.

### 2.2. Data Collection

In this section, all the collection procedure is discussed, which further contain data collection procedures and collection of data delivery.

#### 2.2.1. Data Collection Procedures

*Design of the Questionnaires for Epidemiological Research*. A uniform set of rules for the operation was established. The questionnaire form was first filled out by the subjects. Then, the answers were checked item by item by the specially trained medical staff with the subjects in a face-to-face manner. The survey covered the following dimensions: personal life habits, history of hypertension, history of diabetes, history of myocardial infarction, family history of hypertension, family history of cerebral stroke, smoking history, drinking history, physical activity, sleep duration and quality, educational background, and income. The questionnaire survey was administered by specially trained medical staff following a standard protocol. The measurement methods used in the present study had been described in our previously published paper [8].

The subjects were fasted for 12 h before venous blood collection (5 ml) from the elbow the next morning. The collected blood sample was divided into two tubes. One tube was added with 1 ml of blood sample along with EDTA-K2 anticoagulant. The sample in this tube was used for a routine blood test, which determined the white blood cell count and the platelet count using the ABX fully automated hematology analyzer (ABX MICROS 60 OT Diagnostics). In another tube, 4 ml of the collected blood sample was added and centrifuged. The serum was collected and detected for total cholesterol (TC), triglyceride (TG), high-density lipoprotein cholesterol (HDL-C), low-density lipoprotein cholesterol (LDL-C), and fasting blood glucose (FBG) using Hitachi 7080 Clinical Automatic Chemistry Biochemistry Analyzer. The test operations were undertaken in strict accordance with the kit instructions. Quality control was conducted for each batch of kits. All detections were performed by professionals.

#### 2.2.2. Collection of Delivery Data

The specially trained medical staff filled in the delivery information based on the subjects' self-reported time and place of delivery and their admission records. The following data were collected: age at delivery, delivery time and mode, peripartum blood pressure, height, weight, fundal height, abdominal circumference and edema, fetal gender, fetal body weight and body length, and fetal survival; laboratory tests: platelet count, hemoglobin level, and urine protein; complications in parturients and newborns.

### 2.3. Diagnostic Criteria

#### 2.3.1. Diagnostic Criteria for GH

GH was defined as follows according to the 2015 Guidelines for the Management of Hypertension in Pregnancy [9], having the first experience of high blood pressure after week 20 of pregnancy, with systolic blood pressure (SBP) = 140 mmHg (1 mm Hg = 0.133 KPa) and (or) diastolic blood pressure (DBP) = 90 mm Hg. The subjects recovered from hypertension 12 weeks after delivery.

#### 2.3.2. Definition of CVH Behaviors and Factors

Given the specific situations of Chinese parturients, some modifications of the definition were made based on the one provided by AHA:

1. CVH behaviors includes the following. (1) Smoking status: ① ideal, not smoking at all; ② fair, having once smoked but now quit; ③ poor, still smoking presently. (2) BMI: ① ideal, BMI < 25 kg/m^2^; ② fair, 25∼29.9 kg/m^2^; ③ poor, BMI = 30 kg/m^2^. (3) Physical activity: ① ideal, ≥80 min/week; ② fair, 0–80 min/week; ③ poor, never. (4) Salt intake: ① ideal, preferring bland food; ② fair, neutral; ③ poor, preferring salty food.
2. CVH factors: (1) Total cholesterol: when not taking any lipid-lowering medication. ① Ideal, total cholesterol<5.18 mmol/L; ② fair, total cholesterol 5.18∼6.19 mmol/L, or after having taken some lipid-lowering medication, total cholesterol<5.18 mmol/L; ③ poor, total cholesterol = 6.20 mmol/L; (2) blood pressure: ① ideal, when not taking any antihypertensive medication, systolic blood pressure <120 mm Hg (1 mm Hg = 0.133 kPa) and diastolic blood pressure <80 mm Hg; ② fair, systolic blood pressure 120–139 mm Hg or diastolic blood pressure 80–89 mm Hg, or after having taken antihypertensive medication, blood pressure <120/80 mm Hg; ③ poor, systolic blood pressure = 140 mm Hg or diastolic blood pressure = 90 mm Hg; (3) fasting blood glucose: ① ideal, when not taking any antidiabetic medication, fasting blood glucose <5.6 mmol/L; ② fair, fasting blood glucose 5.6∼7.0 mmol/L; or after having taken antidiabetic medication, fasting blood glucose <5.6 mmol/L; ③ poor, fasting blood glucose = 7.0 mmol/L. CVH scores were assessed according to Mark D. Huffman's simple composite CVH score system [10]. Scores were assigned to the seven CVH metrics according to the following rules: poor = 0 point, fair = 1 point, and ideal = 2 points. The score range was 0–14 points.

### 2.4. Statistical Analysis

The physical examination data of subjects were entered into the computer by specially trained staff at each hospital. The data were transferred via the network to the Oracle Database at the computer room of Kailuan Hospital. The delivery data were then entered into the database using the Excel 2003 software and analyzed by the SPSS 13.0 software. All normally distributed measurement data were expressed as mean ± standard deviation. The data in skewed distribution were first subject to logarithmic transformation and then described statistically. The measurements of the NGH and GH groups were analyzed by the independent samples *t*-test. Ratios were compared by the X^2^ test. *P* < 0.05 (two-sided) was taken to indicate a significant difference.

## 3. Result

### 3.1. General Data of Subjects

A total of 4620 female workers who gave birth at hospitals belonging to Kailuan Medical Group from 1979 to 2012 were preliminarily recruited. After eliminating those with complete data, 4477 subjects were finally included, with an average age of 42.5 ± 9.3. The annual physical examination data of 2012 to 2013 were collected from these subjects. These subjects were divided into the GH group and the NGH group, depending on whether they were combined with GH or not at delivery. It was found that the age at delivery and the age upon the annual physical examination were elder in the GH group than in the NGH group (*P* < 0.05). Upon the annual physical examination, the average levels of BMI, SBP, DBP, FBG, TG, TC, and LDL-C were significantly higher in the GH group than in the NGH group (*P* < 0.05). However, the HDL-C level was significantly lower in the GH group than in the NGH group, see Table 1.

### 3.2. Distribution of Seven CVH Metrics between the NGH and GH Groups

According to the definition of CVH, each of the seven CVH metrics was divided into three levels, namely, ideal, fair, and poor. The statistical analysis showed that the percentage of subjects achieving ideal smoking status in both GH and NG groups was the highest among all seven metrics, while the percentage of subjects achieving the ideal level of physical activity was the lowest in either group. Compared with the NGH group, the percentages of subjects achieving ideal levels of BMI, physical activity, blood pressure, FBG, and cholesterol were significantly lower in the GH group (*P* < 0.05), see Table 2.

### 3.3. The Age Distribution Was Different between the NGH and GH Groups upon the Annual Physical Examination

Therefore, the subjects were stratified by age tertiles into three groups: 23∼≤37 age group, 37∼≤47 age group, and 47∼≤75 age group. The general information of the subjects was further analyzed after age stratification. The results showed that the distributions of age at delivery and the age upon the annual physical examination were not significantly different between GH and NGH subjects from different age groups. In all subjects, the BMI, SBP, DBP, FBG, TG, TC, and LDL-C increased with age, while HDL-C decreased with age. All of the above differences were of statistical significance (*P* < 0.05). The BMI, SBP, DBP, TC, and UA were higher among the younger age subjects with GH than those of subjects without GH from the same age group (*P* < 0.05), see Table 3.

The differences in the distribution of ideal CVH behaviors and factors between NGH and GH groups from different age groups were of statistical significance (*P* < 0.01).

### 3.4. Distribution of CVH Behaviors and Factors in Different Groups Stratified by Age

We found that the percentages of subjects achieving ideal BMI, blood pressure, and FBG decreased with age in both GH and NGH groups (*P* < 0.05). The percentage of subjects with GH achieving ideal BMI in the younger age group (23∼≤37) was lower than that of subjects without GH from the same age group. In the 37∼≤47 age group, the percentage of subjects without GH achieving an ideal level of physical activity was higher than that of subjects with GH, see Table 4 and Figure 1.

## 4. Discussion

Cardiovascular diseases remain the leading cause of death worldwide, and its prevalence has been increasing [11, 12]. AHA has proposed the concept of ideal CVH status to meet Healthy People 2020 goals (to improve the cardiovascular health of the population of the US by 20% and reduce the deaths caused by cardiovascular diseases and stroke by 20%, respectively, by the year 2020). A large number of research studies have focused on the prevalence of ideal CVH behaviors and factors among different populations. Generally speaking, the prevalence of ideal CVH behaviors and factors are very low [13], which in turn has a positive correlation with all-cause mortality [14]. Relevant studies conducted in China have shown that if the Chinese populations can achieve ideal CVH status, about 62.1% of the atherosclerotic cardiovascular events can be prevented, including 38.7% of coronary heart disease events, 66.4% of stroke events, and 60.5% of deaths [15]. At present, experts at home and abroad recommend ideal CVH for primary prevention. The cardiovascular disease continuum begins with GH in females.

In the present study, we tried to identify any differences in the distribution of CVH behaviors and factors in parturients with or without GH. Our study may shed light on future directions in preventing and managing cardiovascular diseases in females.

Our results indicated that regardless of the GH history, the prevalence of ideal CVH behaviors and factors remained low. Whether in the GH or the NGH group, among the seven CVH metrics (including smoking, BMI, physical activity, and salt intake), the percentage of subjects achieving the ideal smoking status was the highest. This result might be due to the fact that we only recruited females. The percentage of subjects with GH achieving an ideal smoking status in the 23∼≤37 age group was lower than that of subjects without GH in the same age group. Whatever the age group, the percentage of subjects achieving an ideal salt intake was below 10%. Moreover, the percentage of subjects achieving an ideal level of physical activity was the lowest in any age group among the seven metrics. The percentage of subjects with GH achieving ideal BMI was lower than that of subjects without GH. Such difference was of statistical significance in the 23∼≤37 age group. Given the above, efforts should be strengthened to increase the percentage of females with a history of GH who achieve an ideal level of physical activity. Particularly, guidance should be provided to young and middle-aged females with a history of GH regarding physical activities, body weight control, and diet to promote their general health.

Upon the annual physical examination, the average levels of SBP, DBP, FBG, TG, TC, and LDL-C were significantly higher in the GH group than in the NGH group (*P* < 0.05). However, the HDL-C level was significantly lower in the GH group than in the NGH group (*P* < 0.05). Moreover, the age distribution was different between the NGH and GH groups upon the annual physical examination. Therefore, the subjects were stratified by age tertiles into three groups: 23∼≤37 age group, 37∼≤47 age group, and 47∼≤75 age group. The general information of the subjects was further analyzed after age stratification. The results showed that the distributions of age at delivery and the age upon the annual physical examination were not significantly different between GH and NGH subjects from different age groups. In all subjects, the SBP, DBP, FBG, TG, TC, and LDL-C increased with age, while HDL-C decreased with age (*P* < 0.05). Among the younger age subjects with GH, the SBP, DBP, TC, and UA were higher than those of subjects without GH from the same age group (*P* < 0.05). Apparently, females with a GH history might be faced with aggregation of cardiovascular risk factors even at a younger age (23∼≤37). Besides, the risk factor indicators were worse than those without a GH history from the same age group. However, such a gap was narrowed with age. It is generally believed that high blood pressure, high blood lipids, and high uric acid are all risk factors for cardiovascular diseases and stroke. Therefore, it is important to help females who have given birth, especially those with a GH history, to control their blood pressure, blood glucose, and blood lipids. Increasing the percentage of these females achieving ideal CVH is vital to prevent cardiovascular diseases in females.

One major highlight of the present study was having confirmed the epidemiological differences in CVH behaviors and factors between females with and without GH history.

### 4.1. Limitation

Our study sheds some light on the early prevention and treatment of cardiovascular diseases in females who have given birth. However, the present study had certain limitations. For example, the salt intake level was self-reported information provided by subjects through the questionnaire survey. We did not determine the 24-h urine sodium level ourselves. Therefore, the applicability of the research findings may be restricted.

## Figures and Tables

**Figure 1:** Distribution of ideal CVH behaviors and factors in different age groups. Note: BMI: body mass index; CVH: cardiovascular health behaviors and factors; GH: gestational hypertension; NGH: nongestational hypertension.

**Table 1:** Comparison of general information among subjects upon physical examination (*x* ± *s*).

Group		NGH group (*n* = 3857)	GH group (*n* = 620)	*P*
Age at delivery (year)		27.1 ± 3.8	27.7 ± 4.5	0.002
Age upon physical examination (year)		41.8 ± 9.07	46.7 ± 9.4	<0.001
Resting heart (beats/min)	Rate	73.27 ± 9.40	72.92 ± 8.76	0.458
BMI (Kg/m^2^)		23.90 ± 3.59	24.93 ± 4.05	<0.001
SBP (mm Hg)		116.75 ± 17.96	125.89 ± 20.32	<0.001
DBP (mm Hg)		76.62 ± 10.18	81.44 ± 10.99	<0.001
FBG (mmol/l)		5.29 ± 1.42	5.55 ± 1.50	<0.001
TG (mmol/l)		1.25 ± 1.16	1.40 ± 1.49	0.015
TC (mmol/l)		4.84 ± 0.97	4.98 ± 1.01	0.003
LDL-C (mmol/l)		2.39 ± 0.97	2.54 ± 0.81	0.001
HDL-C (mmol/l)		1.46 ± 0.47	1.40 ± 0.37	0.006
UA (umol/l)		256.59 ± 65.76	260.60 ± 70.87	0.226

*Note*. BMI (body mass index) = weight (Kg)/height (m^2^); SBP: systolic blood pressure; DBP: diastolic blood pressure; FBG: fasting blood glucose; TG: triglyceride; TC: total cholesterol; LDL-C: low-density lipoprotein cholesterol; DHL-C: high-density density lipoprotein cholesterol; UA: uric acid.

**Table 2:** Distribution of CVH behaviors and factors in NGH and GH groups.

CVH behaviors and group	NGH (*n* = 3857)	GH (*n* = 620)	*χ* ^2^	*P* factors
Smoking	Ideal	3828/99.2	612/98.7	1.890 0.389
	Fair	11/0.3	3/0.5	
	Poor	18/0.5	5/0.8	

BMI	Ideal	2500/64.8	329/53.1	32.885 < 0.001
	Fair	967/25.1	1166/26.0	
	Poor	390/10.1	92/14.8	

Salt intake	Ideal	356/9.2	50/8.1	1.455 0.483
	Fair	3376/87.5	546/88.1	
	Poor	125/3.2	24/3.9	

Physical activity	Ideal	131/3.4	30/4.8	19.963 < 0.001
	Fair	1682/43.6	320/51.8	
	Poor	2044/53.0	270/43.5	

Blood pressure	Ideal	2231/57.8	233/37.6	131.930 < 0.001
	Fair	1177/30.5	222/35.8	
	Poor	449/11.6	165/26.6	

Fasting blood glucose ideal	Ideal	3136/82.0	444/71.6	38.460 < 0.001
	Fair	558/14.5	135/21.8	
	Poor	136/3.5	41/6.6	

Total cholesterol	Ideal	2811/72.9	409/66.0	13.125 0.001
	Fair	776/20.1	161/26.0	
	Poor	270/7.4	50/8.1	

*Note*. BMI: body mass index; CVH: cardiovascular health behaviors and factors; GH: gestational hypertension; NGH: nongestational hypertension.

**Table 3:** Comparison of the general information of subjects stratified by age.

Indicator *P*	23∼37 year old (*n* = 1520)/NGH (*n* = 1400)GH (*n* = 120) *P*			37∼≤47years old (*n* = 1479)/NGH (*n* = 1312) GH ((*n* = 167)			47∼≤75 years old (*n* = 1478)/NGH (*n* = 1145) GH (*n* = 333)		
Age at delivery (year)	26.6 ± 2.5	22.6 ± 2.6	0.874	26.3 ± 3.4	27.0 ± 4.4	0.012	28.4 ± 4.9	28.7 ± 5.0	0.001
Age upon physical examination (year)	32.1 ± 2.9	32.3 ± 2.5	0.381	42.6 ± 2.7	42.8 ± 2.7	0.509	52.8 ± 4.5	53.8 ± 5.0	0.296
Resting heart rate (beats/min)	73.26 ± 9.41	73.31 ± 10.17	0.961	72.25 ± 8.31	72.95 ± 8.44	0.366	72.77 ± 8.41	74.43 ± 10.34	0.022
BMI (Kg/m^2^)	22.86 ± 3.53	23.94 ± 4.95	0.04	23.73 ± 3.25	24.65 ± 4.38	0.003	25.20 ± 3.64	25.42 ± 3.41	0.364
SBP (mm Hg)	107.79 ± 11.48	113.34 ± 13.18	<0.001	114.28 ± 14.18	121.39 ± 17.69	<0.001	128.56 ± 20.46	132.7 ± 20.9	<0.001
DBP (mm Hg)	71.84 ± 7.86	76.03 ± 9.58	<0.001	75.98 ± 8.9	80.66 ± 10.35	<0.001	82.18 ± 10.84	83.82 ± 11.05	0.01
FBG (mmol/l)	5.00 ± 1.34	5.13 ± 0.64	0.29	5.24 ± 1.19	5.39 ± 1.57	0.17	5.68 ± 1.63	5.80 ± 1.62	0.262
TG (mmol/l)	1.00 ± 0.67	1.45 ± 2.83	<0.001	1.22 ± 1.24	1.27 ± 0.93	0.639	1.60 ± 1.40	1.67 ± 1.91	0.125
TC (mmol/l)	4.57 ± 0.89	4.79 ± 1.01	0.012	4.80 ± 0.94	4.74 ± 0.89	0.44	5.2 ± 0.98	5.14 ± 0.98	0.617
LDL-C (mmol/l)	2.25 ± 0.81	2.34 ± 0.91	0.294	2.32 ± 0.82	2.42 ± 0.73	0.182	2.63 ± 1.22	2.69 ± 0.78	0.465
HDL-C (mmol/l)	1.49 ± 0.61	1.40 ± 0.35	0.158	1.48 ± 0.37	1.39 ± 0.31	0.012	1.41 ± 0.37	1.41 ± 0.41	0.763
UA (umol/l)	262.17 ± 65.50	291.65 ± 80.47	<0.001	250.51 ± 65.82	247.79 ± 64.32	0.656	292.11 ± 67.83	293.09 ± 66.12	0.65

*Note*. BMI (body mass index) = weight (Kg)/height(m)^2^; SBP: systolic blood pressure; DBP: diastolic blood pressure; FBG: fasting blood glucose; TG: triglyceride; TC: total cholesterol; LDL-C: low-density lipoprotein cholesterol; DHL-C: high-density density lipoprotein cholesterol; UA: uric acid.

**Table 4:** Distribution of CVH behaviors and factors in different age groups.

		23∼37 year old (*n* = 1520)/		37∼≤47 years old (*n* = 1479)			47∼≤75 years old (*n* = 1478)				
		NGH (*n* = 1400)	GH (*n* = 120)	NGH (*n* = 1312)	GH (*n* = 167)		NGH (*n* = 1145)				GH (*n* = 333)
Metrics	Gender										
Smoking	Ideal (*n*/%)	1395/99.6	118/98.3	1301/99.2	166/99.4		1132/98.9			328/98.5	
	Fair (*n*/%)	1/0.1	1/0.8	3/0.2	1/0.6		7/0.6		1/0.3		
	Poor (*n*/%)	4/0.3	1/0.8	8/0.6 0/0			6/0.5		4/1.2		
		*χ* ^2^ = 5.903	*P*=0.052	*χ* ^2^ = 1.770		*P*=0.413	*χ* ^2^ = 2.213		*P*=0.331		

BMI	Ideal (*n*/%)	1072/76.6	79/65.8	861/65.6		99/59.3	567/49.5		151/45.3		
	Fair (*n*/%)	232/16.6	29/24.2	345/26.3		47/28.1	390/34.1		123/36.9		
	Poor (*n*/%)	96/6.9	12/10.0	106/8.1		21/12.6	188/16.4 59/17.7				
		*χ* ^2^ = 6.033	*P*=0.031	*χ* ^2^ = 4.596		*P*=0.100	*χ* ^2^ = 1.800		*P*=0.407		

Salt intake	Ideal (*n*/%)	160/11.4	9/7.5	139/10.6		24/14.4	57/5.0		50/8.1		
	Fair (*n*/%)	1167/83.4 101/84.2		1136/86.6		135/80.8	1073/93.7		546/88.1		
	Poor (*n*/%)	73/5.2	10/8.3	37/2.8		8/4.8	15/1.3	24/3.9			
		*χ* ^2^ = 3.512	*P*=0.173	*χ* ^2^ = 4.377		*P*=0.112	*χ* ^2^ = 0.458	*P*=0.795			

Physical activity	Ideal (*n*/%)	6/5.0	30/2.1	56/4.3		8/4.8	45/3.9	16/4.8			
	Fair (*n*/%)	562/40.1	54/45.0	545/41.5		89/53.3	575/50.2	177/53.2			
	Poor (*n*/%)	808/57.7	60/50.9	711/54.2		70/41.9	525/45.9	140/42.0			
		*χ* ^2^ = 5.605	*P*=0.061	*χ* ^2^ = 9.095		*P*=0.011	*χ* ^2^ = 1.747	*P*=0.417			
Blood pressure	Ideal (n/%)	65/54.2	1061/75.8	774/59.0		68/40.7	396/34.6	100/30.0			
	Fair (n/%)	310/22.1	45/37.5	438/33.4		68/40.7	429/37.5	109/32.7			
	Poor (n/%)	29/2.1	10/8.3	100/7.6		31/18.6	320/27.9	124/37.2			
		*χ* ^2^ = 35.025	*P* < 0.001	*χ* ^2^ = 31.041		*P* < 0.001	*χ* ^2^ = 10.594	*P*=0.005			

Fasting blood glucose	Ideal (*n*/%)	99/82.5	1286/91.9	1085/82.7		128/76.6	792/69.2	217/65.2			
	Fair (*n*/%)	105/7.5	19/15.8	193/14.7		35/21.0	260/22.7	81/24.3			
	Poor (*n*/%)	9/0.6	2/1.7	34/2.6		4/2.4	93/8.1 5	35/10.			
		*χ* ^2^ = 12.072	*P*=0.002	*χ* ^2^ = 4.435		*P*=0.109	*χ* ^2^ = 2.598	*P*=0.273			

Total cholesterol	Ideal (*n*/%)	89/74.2	1161/82.9	983/74.9		128/76.6	667/58.3	192/57.7			
	Fair (*n*/%)	190/13.6	25/20.8	254/19.4		33/19.8	332/29.0	103/30.9			
	Poor (*n*/%)	49/3.5	6/5.0	75/5.7		6/6.0	146/12.8	38/11.4			
		*χ* ^2^ = 5.840	*P* = 0.054	*χ* ^2^ = 1.291		*P* = 0.524	*χ* ^2^ = 0.716	*P*=0.699			

*Note*. BMI: body mass index; CVH: cardiovascular health behaviors and factors; GH: gestational hypertension; NGH: nongestational hypertension.

## Data Availability

The simulation experiment data used to support the findings of this study are available from the corresponding author upon request.
